The article "Analysis of Effect of Six Sigma Method Combined with CI Strategy on Improving of Nursing Quality in Outpatient Infusion Rooms" was retracted in 2023. Reasons: unreliable results or conclusions; concerns about the data; concerns about the peer review; concerns about the citations.

# Analysis of Effect of Six Sigma Method Combined with CI Strategy on Improving of Nursing Quality in Outpatient Infusion Rooms

**DOI:** 10.1155/2022/8975435

**Published:** 2022-10-08

**Authors:** Xiuqin Shen, Jiao Wei, Ying Zhang, Yinying Zhang

**Affiliations:** Department of Infusion Center, The First Affiliated Hospital of Soochow University, Suzhou, Jiangsu 215000, China

## Abstract

**Objective:**

The infusion room is the last part of an outpatient visit, with high patient density, large staff mobility, and a wide variety of conditions. In addition, most patients are accompanied by their families during infusion, and nursing staff in infusion rooms have to face more trivial and miscellaneous tasks than nursing staff in other treatment departments, which are more complex. The purpose of this research is to explore the impact of the Six Sigma method and CI strategy on the quality of nursing management in infusion rooms, so as to provide reference for clinical research.

**Methods:**

A total of 2142 patients treated in our outpatient infusion rooms from June 2019 to June 2020 was included into this retrospective analysis. Of these, 1105 patients admitted before 2020 received routine care management services and were considered as the control group. Another 1037 patients were admitted after 2020 and received the Six Sigma method combined with CI strategic care management and were considered as the research group. The incidence of adverse events during treatment was counted in both groups, and patients' compliance behavior and psychology were investigated. After treatment, patients' evaluation of the quality of nursing and their satisfaction with the nursing were investigated.

**Results:**

The incidence of adverse events during infusion in the research group was dramatically lower than that in the control group, while the compliance behavior scores were higher (*P* < 0.05). In addition, SAS and SDS in the research group were lower than those in the control group, while the quality of nursing were higher (*P* < 0.05). It was also clear that the research group had 93.39% satisfaction with nursing, which was also higher than the control group (*P* < 0.05).

**Conclusion:**

Implementation of infusion room nursing management according to the Six Sigma method with CI strategic plan can avoid adverse events and improve infusion nursing satisfaction. It also helps reduce the incidence of dispute events.

## 1. Introduction

The infusion room is the last part of an outpatient visit, with high patient density, large staff mobility, and a wide variety of conditions. In addition, most patients are accompanied by their families during infusion, and nursing staff in infusion rooms have to face more trivial and miscellaneous tasks than nursing staff in other treatment departments, which are more complex [1]. As a result, nursing in infusion rooms is more intensive and disorganized [2]. Surveys have shown that in tertiary hospitals, the average daily outpatient infusion room receives more than about 300 patients alone. With the addition of patients' accompanying persons or family members, the average daily population flow in the infusion room is basically at 500-800 visits/day [3]. At the same time, patients are characterized by limited mobility, organic discomfort, and emotional agitation during infusion. Accompanying family members are prone to adverse emotions due to the limited things they can undertake, which makes it further difficult to carry out nursing work [4]. Infusion room nursing has the risk of different degrees and aspects of adverse events that affect the quality of nursing under multiple factors, and nursing management is an effective way to improve the quality and efficiency of nursing [5].

Nursing service strategies in outpatient infusion rooms need to meet both broad applicability and must be time-effective and can be completed within a limited working time [6]. Among the nursing management programs, the Six Sigma method is considered a near perfect quality management program, proposed for Bill Smith of Motorola [7]. This management scheme applied to nursing management can clearly point out the problems in nursing and develop appropriate solutions [8]. Recently, Six Sigma has also been gradually gaining attention in clinical healthcare services and has now achieved excellent results in clinical departments such as the operating room and ophthalmology [9, 10]. Corporate Identity (CI) strategy is mostly used in “corporate image” management, but with the awakening of hospitals to their own brand and image awareness and attention, some studies have also incorporated CI strategy ideas into nursing management and achieved more desirable results; For example, Hardy et al. proposed that the CI strategy is the best management choice for the future clinical radiology department [11, 12]; Becze stated that the CI strategy will be a necessary measure for the future hospital [13]. We believe that the Six Sigma method and CI strategy are equally effective in improving the overall quality of nursing and patient treatment experience in outpatient infusion rooms and reducing the occurrence of doctor-patient disputes, but there are no studies at home or abroad to confirm this view.

Since 2020, our hospital has been carrying out the nursing management of the Six Sigma method and CI strategic thinking in infusion rooms, and sufficient cases have been accumulated so far. So, a retrospective analysis will be performed. Our purpose is to find a management solution suitable for outpatient infusion rooms, which can improve the quality of nursing services while reducing the pressure of nursing work. This has extremely important reference significance for outpatient infusion rooms in all hospitals around the world in the future.

## 2. Materials and Methods

### 2.1. General Data

The infusion rooms in our hospital were regarded as the study site, and patients receiving infusion therapy were included as subjects. They were divided into the control group (1105 cases, included from June to December 2019) and the research group (1037 cases, included from January to June 2020) based on the time of inclusion. In the control group, there were 539 males (48.78%) and 566 females (51.22%), with an average age of 41.92 ± 15.37 years. In the research group, there were 507 males (48.89%) and 530 females (51.11%), with an average age of 42.06 ± 16.12 years. Among them, patients in the control group received conventional infusion room nursing management, and the research group received the Six Sigma method combined with CI strategic nursing management. This study has been approved by the Ethics Committee of our hospital, and all research subjects signed the informed consent form.

### 2.2. Inclusion and Exclusion Criteria

Inclusion criteria are as follows: (1) receiving infusion therapy in infusion rooms after a visit to our hospital; (2) being watched by father or mother, partner, or child; (3) Age: 18-75 years old; (4) basic reading and writing skills; and (5) signed informed consent forms. Exclusion criteria are as follows: (1) receiving nursing interventions from nondesignated caregivers, (2) combined audiovisual dysfunction, (3) not having basic reading and writing skills, and (4) no family or caregiver care.

### 2.3. Methods

Nursing services are completed by the same nursing team in our hospital, and all nurses have 3-5 years of work experience. Control group: routine nursing management was implemented. Nursing staff are required to carefully check identification information, prescription, and drug information before performing infusion operations, to develop infusion nursing operation procedures, and to link the quality of infusion room nursing to nurse performance, etc. Research group: Six Sigma method in conjunction with CI strategic nursing management was performed. Combining the definition, measurement, analysis, improvement, and control phases of the Six Sigma method with the mind identification (MI), behavioral identity (BI), and visual identity (VI) of the CI strategy, this research nursing management program was developed: (1) Definition phase: the proportion of adverse events of patients in infusion nursing and their satisfaction were seen as criteria to assess the quality of nursing management, to reduce the incidence of adverse events in infusion and increase satisfaction and improve the quality of nursing management. (2) Analysis phase: synthesizing our previous nursing experience with relevant literature [13–15], we concluded that the main reasons for adverse reactions and dissatisfaction with nursing expressed by patients during infusion can be divided into two areas. On the one hand, the performance of nursing staff does not meet the clinical requirements, such as not paying attention to the hygienic environment or having a lazy mentality leading to the lack of classification of medical and domestic waste, the lack of skill in infusion operation leading to repeated punctures and irregular fixation of dressings, and the low cooperation between nurses leading to long waiting time for infusion for patients. On the other hand, patients and their accompanying family members have insufficient knowledge of infusion rooms and the requirements related to infusion treatment, such as lack of knowledge of garbage sorting leading to difficulties in sanitary management of the rooms, and precautions after infusion bringing about needle dislodgement and serious bleeding back. Therefore, the focus of implementing quality of nursing management for patients in the 2020 group can be determined to include both nursing staff management and patient cognitive management. (3) Improvement phase: CI strategies were integrated into this phase. ① Build professional beliefs for nursing staff through culture building. Create a good nursing atmosphere, such as posting slogans in the infusion rooms with the themes of “Respect for Life” and “High-quality Nursing.” Regularly organize nursing staff to carry out cultural performances with the theme of “ethics of nursing behavior” and encourage nursing staff to promote nursing cultural quality by adapting songs, creating skits, writing stand-up comedy, etc. in conjunction with their own clinical work experience. ② Implement nursing behavior management for nursing staff. First, professional nursing skills training was implemented regularly for nursing staff to improve their professional competence. In the process of training, nurses should improve their awareness of self-protection, especially when separating used needles to avoid needle-stick injuries. Then, we formulate the duties of nursing staff in infusion rooms, including the hygienic management of infusion rooms (such as waste classification, ventilation management, and infrastructure disinfection), standardization of the infusion care process, and the preservation program for disposable sterile medical supplies. Subsequently, a code of ethical conduct for nursing staff was written, stipulating that nursing staff should use honorific form and be gentle when dealing with patients and their families, and should not show perfunctory emotions in response to repeated inquiries from patients. Meantime, nursing staff were trained in communication skills so that they could implement infusion-related health education to patients as briefly, quickly, and effectively as possible (e.g., no excessive movement of the limb on the receiving side during infusion, personal garbage needs to be disposed of in a fixed garbage can, no loud noises are allowed during infusion unless necessary, and nursing staff should be informed immediately of any discomfort). ③ Standardize the visual image of nursing staff. Regularly issue new work clothes to nursing staff to ensure that they are well dressed and clean. Issue each caregiver a badge with his or her name and require it to be worn daily. We also standardize the accessories and makeup of nursing staff so that their external appearance remains gentle and approachable. (5) Control stage: develop quality assessment indexes according to the nursing program, clarify the work requirements for nursing staff at all levels, regularly inspect the work of nursing staff, and link the inspection results to their performance.

### 2.4. Outcome Measures

1. The occurrence of adverse events such as inadequate sanitary management, inadequate management of medical items, infusion operation errors and unsuccessful completion of infusion in the infusion rooms during the study period was counted, and the incidence of adverse events was calculated
2. Compliance behavior: before the end of treatment, the compliance behavior of patients and family members during infusion was assessed by a departmental compliance questionnaire distributed by nurses [16]. It includes 4 items of wandering infusion, patient hygiene behavior, family hygiene behavior, and family caregiving behavior. Each item has 25 points out of 100, the higher the score, the higher the degree of compliance behavior
3. Psychology: after treatment, patients' psychology was assessed using the Self-Rating Scale for Anxiety (SAS) and Depression (SDS) [17], the scoring results are from 0 to 100 points, with higher scores indicating more severe negative feelings of anxiety and depression
4. Nursing quality evaluation: a survey was conducted using a nursing quality questionnaire [18]. It contained four aspects: technical level, infusion environment, etiquette service, and psychological guidance, each of which was scored out of 10. The total score was calculated; the higher the score, the higher the nursing quality
5. Nursing satisfaction: a self-administered nursing satisfaction questionnaire was developed [19], which assessed six items including infusion room environment, nursing intervention during waiting for infusion, service attitude, infusion technique level, communication, postinfusion precautions explanation, and overall satisfaction; each item was set as three options of very satisfied, satisfied, and dissatisfied. In the meantime, patients were asked to indicate the reason for dissatisfaction after selecting the dissatisfaction option. Total satisfaction rate = (very satisfied + satisfied)/total × 100%. Both quality of care and satisfaction surveys were conducted when patients completed treatment and were ready to leave the hospital

### 2.5. Statistical Analysis

Data were entered into SPSS 22.0, and the counting data such as the incidence of adverse events, nursing satisfaction rate, and gender were expressed by (*n* (%)) with a *χ*^2^ test. Age was expressed as $\bar{x}\pm s$, *t*-test was performed, and statistical differences were represented as *P* < 0.05.

## 3. Results

### 3.1. Comparison of General Data

Comparing the general data of gender, age, and marital status between the two groups, we found that the differences in gender, age, marital status, and primary caregiver were not statistically remarkable (*P* > 0.05, Table 1), confirming comparability between both groups.

### 3.2. Comparison of Incidence of Adverse Events between Both Groups

Subsequently, the total rate of adverse events in the research group was only 6.56%, which was dramatically lower compared to the control group (13.48%) (*P* < 0.001). It was also seen that the incidence of adverse events such as inadequate hygiene management, improper management of medical items, infusion operation errors, and unsuccessful completion of infusion were all lower in the research group than in the control group (*P* < 0.05, Table 2).

### 3.3. Comparison of Compliance Behavior Scores between Both Groups

The results of compliance behavior scores in both groups denoted that the total score of the research group (23.14 ± 2.65) was higher than that of the control group (17.15 ± 3.91) (*P* < 0.05, Figure 1(a)). It was also seen that the research group also had higher score results than the control group in all domains of wandering infusion, patient hygiene behavior, family hygiene behavior, and family caregiving behavior (*P* < 0.05, Figures 1(b)–1(e)).

### 3.4. Comparison of Psychology between Both Groups

The SAS score of the research group was 37.07 ± 17.88, which was lower than that of the control group (*P* < 0.05, Figure 2(a)). Besides, the SDS score in the research group was 31.79 ± 17.44, which was also dramatically lower than that in the control group (*P* < 0.05, Figure 2(b)).

### 3.5. Comparison of Quality of Nursing Evaluation between Both Groups

The ratings of nursing staff technical level, infusion environment, etiquette service, and psychological guidance in the research group were 9.15 ± 0.72, 9.13 ± 0.65, 8.86 ± 0.86, and 8.76 ± 1.23, respectively. Compared with the control group, the evaluation scores of technical level, infusion environment, etiquette service, and psychological guidance were higher in the research group (*P* < 0.05, Figures 3(a)–3(d)). The research group was also higher than the control group when compared with the total quality of nursing evaluation score of both groups (*P* < 0.05, Figure 3(e)).

### 3.6. Comparison of Nursing Satisfaction between Both Groups

The nursing satisfaction survey of both groups manifested that the total satisfaction rate of the research group was 93.39%, which was higher than that of the control group (90.21%) (*P* = 0.017, Table 3).

## 4. Discussion

Six Sigma is one of the quality management methods, which was first applied in the quality management of manufacturing companies and gradually expanded to the quality management of the service industry through subsequent development [20]. Nursing interventions are among the service interventions. Research has shown that adding the Six Sigma management model to the management of hospital service quality allows for an increase in the scientific nature of hospital care management and an increase in patient satisfaction [21]. Previous studies have shown that performing Six Sigma quality of nursing management in the labor and delivery office has been shown to promote standardized writing of nursing documents and cognitive education of nursing knowledge [22].

The infusion room is a separate clinic for intravenous treatment in the hospital, and the work is mainly carried out by nursing staff, so the quality of nursing is the main reflection of the quality of management in the room. In the case of emergency infusion rooms, the implementation of nursing management in conjunction with the Six Sigma method can reduce the risk of dispute events while improving patient satisfaction [23]. CI strategy is mostly applied to the construction of corporate culture, through the planning and improvement of corporate image, to achieve the ultimate goal of deepening the quality image of the company into the minds of the public [24]. Previous studies related to the integration of CI strategies into nursing quality management (especially nursing quality management in infusion rooms) are fewer, which researchers believe is related to the fact that most researchers have focused more on nursing operations and nursing technology in their studies to the neglect of nursing environment and nursing culture construction [25]. Therefore, in this study, while applying the Six Sigma method to improve the quality of nursing management in infusion rooms, CI strategic thinking was incorporated into it in the hope that the quality of nursing in infusion rooms of our hospital could be optimized in terms of both actual nursing work and nursing thinking.

This study demonstrated that the incidence of adverse events such as inadequate hygienic management during infusion, improper management of medical items, infusion operation errors, and unsuccessful completion of infusion were lower in the research group than in the control group. It is evident that the implementation of the new care management policy has improved the safety of care in all aspects and the improvement is holistic in nature. There are reasons as follows: (1) To solve the problem completely, we need to identify the root causes of the problems. The Six Sigma management process, inquiring about nursing adverse events and analyzing the causative factors as a key step, has a directive effect on the direction of subsequent nursing and also allows for more targeted nursing interventions [26]. (2) CI strategic thinking is not a fetter and supervision of nursing staff, but a correct guidance of nursing concepts and ideas. Positive, conscientious, and dedicated nursing thinking can increase the patience of nursing staff for their own work and the acceptance of patients and their families. In turn, the nursing staff will be able to think more clearly in the boring, busy, and messy infusion room nursing work [27]. Moreover, we also found that the compliance behavior of the research group was dramatically improved, while the poor psychology was improved. Research has noted that most patients feel they are not being given enough attention due to the large number of people in infusion rooms, the noisy environment, and the high turnover of staff [28]. At the same time, patients generally exhibit resistance and rejection of health care workers due to the pain caused by the disease [29]. This not only greatly increases the incidence of doctor-patient disputes but also will seriously affect nursing treatment. And the results of this experiment revealed that the use of the Six Sigma method and CI strategic thinking for nursing management can effectively compensate for this shortcoming, reduce patients' resistance to health care workers, and improve treatment acceptance. It was seen that patients in the research group rated the quality of nursing and were more satisfied with it than the control group. There are reasons as follows: (1) A reduction in the incidence of adverse events reduces the tension of patients and their families and leads to an increase in their satisfaction. (2) The first step in six sigma is to set goals. The goal in this study was to improve patient satisfaction with nursing, and the motivation of nursing staff was improved by linking quality of nursing to salary performance after clarifying the goals of nursing management [30]. (3) The CI strategy implements planning and management of the nursing staff's external appearance and internal temperament, making it easier for patients to accept the nursing staff and follow their advice. An increase in nursing satisfaction increases patients' trust in nursing staff and improves their compliance with nursing operations, so patients and their families show increased performance in support of nursing.

At present, the Six Sigma method in nursing management has received some attention and application, but CI strategic thinking is still relatively rare, which still deserves further exploration. Furthermore, the basis for the grouping in this study was related to different approaches to nursing management on the one hand and to time years on the other, which may also produce potential factors affecting the results. Thus, we still need to follow up with a clinical randomized controlled trial to further confirm the effectiveness of the application of the Six Sigma method with the CI strategic plan to implement infusion room nursing management. In addition, in modern infusion room nursing management, we need to pay attention not only to the performance and operational skills of nursing staff but also to the construction of the nursing environment. We can further optimize the environment of infusion rooms to enhance the treatment experience of patients.

## 5. Conclusion

Implementation of infusion room nursing management based on the Six Sigma method with CI strategic plan can avoid adverse events and improve infusion nursing satisfaction. It can help reduce the incidence of dispute events.

## Figures and Tables

**Figure 1:** Comparison of compliance behavior scores between both groups. (a) Comparison of total compliance behavior scores. (b) Comparison of wandering infusion field scores. (c) Comparison of patient health behavior domain scores. (d) Comparison of family members' hygiene behavior scores. (e) Comparison of family caregiving behavior domain scores. ^∗∗∗^*P* < 0.001.

**Figure 2:** Comparison of mental scores between both groups. (a) Comparison of SAS score results. (b) Comparison of SDS score results. ^∗^*P* < 0.05.

**Figure 3:** Comparison of quality of nursing evaluation between both groups. (a) Comparison of nursing staff skill level evaluation results. (b) Comparison of infusion environment evaluation results. (c) Comparison of etiquette services evaluation results. (d) Comparison of psychological guidance evaluation results. (e) Comparison of total quality of nursing evaluation scores. ^∗∗^*P* < 0.01.

**Table 1:** Comparison of general data between both groups ($\bar{x}\pm s$/*n* (%)).

Groups	Cases	Gender		Age (year)	Marital status				Primary caregiver		
		Male	Female		Unmarried	Married	Divorced	Widowed	Man and wife	Parents	Children
Control group	1105	539 (48.78)	566 (51.22)	41.92 ± 15.37	230 (20.81)	571 (51.67)	149 (13.48)	155 (14.03)	514 (46.52)	377 (34.12)	214 (19.37)
Research group	1037	507 (48.89)	530 (51.11)	42.06 ± 16.12	225 (21.70)	519 (50.05)	128 (12.34)	165 (15.91)	495 (47.73)	371 (35.78)	171 (16.49)
*t*/*χ*^2^		0.003		0.206	0.249	0.566	0.618	1494	0.319	2.971	3.003
*P*		0.958		0.837	0.618	0.452	0.432	0.222	0.572	0.082	0.083

**Table 2:** Comparison of incidence of adverse events between both groups (*n* (%)).

Adverse events	Performance	Control group (*n* = 1105)	Research group (*n* = 1037)	*χ* ^2^	*P*
Inadequate hygiene management	Uncategorized garbage	13 (1.18)	6 (0.58)		
	Incomplete cleaning and disinfection records	22 (1.99)	13 (1.25)		
	Total	35 (3.17)	19 (1.83)	3.881	0.049

Improper management of medical items	Expired sterile infusion items	3 (0.27)	0 (0.00)		
	Contamination of sterile infusion items	2 (0.18)	0 (0.00)		
	Total	5 (0.45)	0(0.00)	4.682	0.030

Infusion operation errors	Incorrect patient information verification	3 (0.27)	0 (0.00)		
	Wrong configuration of drug solution	3 (0.27)	0 (0.00)		
	Repeated punctures	11 (1.00)	5 (0.48)		
	Drug extravasation	9 (0.81)	4 (0.39)		
	Irregular fixation of dressing	26 (2.35)	14 (1.35)		
	Total	52 (4.71)	23 (2.22)	9.800	0.002

Unsuccessful completion of infusion	Needle blockage	10 (0.90)	3 (0.29)		
	Localized redness and swelling at the puncture site	8 (0.72)	3 (0.29)		
	Severe hemorrhage	31 (2.81)	18 (1.74)		
	Needle dislodged	8 (0.72)	2 (0.19)		
	Total	57 (5.16)	26 (2.51)	10.095	0.001

Total		149 (13.48)	68 (6.56)	28.192	<0.001

**Table 3:** Comparison of both groups' satisfaction with nursing (*n* (%)).

Groups	Cases	Very satisfied	Satisfied	Dissatisfied	Total satisfaction rate
Control group	1083	226 (20.87)	751 (69.34)	106 (9.79)	977 (90.21)
Research group	998	298 (29.86)	634 (63.53)	66 (6.61)	932 (93.39)
*χ* ^2^					5.661
*P*					0.017

## Data Availability

The data used in the article is obtained from the corresponding author upon reasonable request.
